The article "Geniposide Alleviates Oxidative Stress of Mice With Depression-Like Behaviors by Upregulating Six3os1" was retracted in 2026. Reasons: original data or images not available; concerns about the images.

# Geniposide Alleviates Oxidative Stress of Mice With Depression-Like Behaviors by Upregulating Six3os1

**DOI:** 10.3389/fcell.2020.553728

**Published:** 2020-10-22

**Authors:** Tianyu Zou, Kazuo Sugimoto, Jielin Zhang, Yongxiu Liu, Yiming Zhang, Hao Liang, Yinan Jiang, Jing Wang, Guoxiang Duan, Cheng Mei

**Affiliations:** ^1^Department of Encephalopathy, Heilongjiang Academy of Medical Sciences, Harbin, China; ^2^Department of Neurology, Dongzhimen Hospital, Beijing University of Chinese Medicine, Beijing, China; ^3^Department of Dermatology, Heilongjiang Provincial Hospital Affiliated to Harbin Institute of Technology, Harbin, China

**Keywords:** depression, geniposide, Six3os1, miR-511-3p, FEZF1, Akt signaling pathway, oxidative stress 3

## Abstract

Depression is a major cause of disease burden and severely impairs well-being of patients around the globe. Geniposide (GP) has been revealed to play a significant role in depression treatment. Of note, RNA sequencing of this study identified highly expressed long non-coding RNA Six3os1 in response to GP treatment. Thus, we aim to explore how GP affected chronic unpredictable mild stress (CUMS)-induced depression-like behaviors in mice *in vivo* and *in vitro* and the downstream molecular mechanism related to Six3os1. The relationship of Six3os1, miR-511-3p and Fezf1 was evaluated by dual-luciferase reporter gene assay, RIP assay, and RNA pulling down assay. Ectopic expression and knockdown experiments were developed in CUMS-induced mice and neurons with or without GP treatment. *In vitro* experiments and behavioral tests were conducted to examine alteration of CUMS-triggered oxidative stress following different interferences. The experimental data validated that GP treatment resulted in high expression of Six3os1 and Fezf1 and poor expression of miR-511-3p in CUMS-induced neurons. Six3os1 activated the AKT signaling pathway by upregulating miR-511-3p-targeted Fezf1. Either GP treatment or overexpression of Six3os1 or Fezf1 alleviated depression-like behaviors of CUMS-induced mice. GP treatment, miR-511-3p inhibition or overexpression of Six3os1 or Fezf1 not only reduced oxidative stress in CUMS-induced mice and neurons, but also reduced CUMS-induced neuronal apoptosis. Collectively, GP treatment-mediated Six3os1 upregulation ameliorated oxidative stress of mice with depression-like behaviors *via* the miR-511-3p/Fezf1/AKT axis.

## Introduction

Depression is considered as a prevalent neuropsychiatric disorder, affecting over 300 million people around the world (Kenning et al., 2019). The main risk factors contributing to depression include financial problems, inferior social status, female sex, stress events in life, chronic or severe diseases, dietary dysfunction, and deficiency of Vitamin D (Razzak et al., 2019). Although computer-based psychological therapies have some efficacy in treating depression (Richards and Richardson, 2012), there is an urgent need for new effective and novel therapeutic approaches for depression (Johansson et al., 2019). Moreover, the neurobiology of depression is accompanied by oxidative stress in the brain and throughout the organism (Silva et al., 2016). In terms of the chronic unpredictable mild stress (CUMS)-induced depression, traditional Chinese medicine has been applied for controlling CUMS-induced depression-like behaviors (Qu et al., 2019). Therefore, it is necessary to explore the specific mechanism of traditional Chinese medicine in CUMS-induced depression-like behaviors.

Geniposide (GP), a bioactive iridoid glycoside isolated from *Gardenia jasminoides* Ellis and as an agonist of Glucagon-like peptide-1 receptor (GLP-1R), was revealed to display an anti-depression role in rodent models (Zhao Y. et al., 2018). Importantly, CUMS-induced depression-like behaviors in rats could be affected via modulation of the hypothalamus/pituitary/adrenal axis (Cai et al., 2015). Previous work has clearly highlighted the important roles of long non-coding RNAs (LncRNAs or lncRNAs) in neuron function, neurodegenerative diseases and brain development (Wu et al., 2013). For example, lncRNA Six3os exerted effects on neural development in the retina by regulating Six3 activity (Rapicavoli et al., 2011). Additionally, microRNAs (miRNAs) are emerging as a potential treatment strategy for depression due to its capacity in influencing neuronal physiology (Hansen and Obrietan, 2013). In human beings, miR-511 was found to be highly expressed as compared with controls in dead basolateral amygdala from suicided individuals due to depressive attack (Maheu et al., 2015). Notably, another lncRNA prognosis-associated gallbladder cancer competitively bound to miR-511 in both hyperresponsiveness and human gallbladder cancer has been previously highlighted (Wu et al., 2017; Li et al., 2018), which indicated that miR-511 could be regulated by lncRNAs.

Previous studies have reported that the Fez family zinc finger protein 1 (Fezf1) serves as an important transcription factor to mediate neurological development (Shimizu et al., 2010; Lan et al., 2018). Furthermore, Fezf1 regulated various cell processes in glioma cells by activating the AKT-ERK signaling pathway (Yu et al., 2018). Meanwhile the PI3K/AKT/FoxO1 pathway is implicated in the mechanism of action of the flavone baicalin in alleviating depression-like behaviors by suppressing the Toll-like receptor TLR4 (Guo et al., 2019). Moreover, miR-511 significantly accelerated procine kidney (PK-15) cell apoptosis by reducing the extent of AKT phosphorylation (Wei et al., 2019). Herein, from the aforementioned findings, we might hypothesize that GP could affect the progression of CUMS-induced depression by mediating Six3os1, acting in association with regulation of the miR-511-3p/Fezf1/AKT axis. Therefore, we undertook a series of experiments in the CUMS model aiming at illuminating this pathway as a potential target for a more efficacious personalized treatment for depression.

## Materials and Methods

### Ethics Statement

The animal use and experimental procedures in this study were conducted in accordance with the Guide for the Care and Use of Laboratory Animals published by the National Institutes of Health. The animal experiments were approved by the animal ethics committee of Heilongjiang Academy of Chinese Medical Sciences (approved protocol number: 201910021).

### Drugs and Chemicals

GP (99.52% purity) purchased from MedChemExpress Co., Ltd (HY-N0009, Med New Jersey, United States) (Supplementary Figure S1) was dissolved in dimethyl sulfoxide (DMSO) (D2650, Sigma-Aldrich Chemical Company, St Louis, MO, United States). In animal experiments, GP was diluted with DMSO to different concentrations of 25, 50, and 100 mg/kg (Cai et al., 2015); meanwhile, a stock solution at the concentration of 10 μM (Liu et al., 2017) was used and stored at −80°C.

Other chemicals are listed as follows: sodium pyruvate (11360070, Gibco, United States); 2-[4-(2-Hydroxyethyl)-1-piperazinyl] ethanesulfonic acid (HEPES, 15630080, Gibco, Carlsbad, CA, United States); Hank’s balanced salt solution (HBSS, 14170112, Gibco, United States); Dulbecco’s Modified Eagle Medium (DMEM) (10569044, Gibco, United States); Neurobasal medium (21103049, Gibco, United States); B-27 (17504044, Gibco, United States); L-glutamine (25030081, Gibco, United States); streptomycin (15070063); poly-D-lysine (PDL, A3890401, Gibco, United States); trypsin (25200056, Gibco, United States); Trizol (16096020, Thermo Fisher Scientific Inc., Waltham, MA, United States); electrochemiluminescence (ECL) (#1705062, Bio-Rad, Inc., Hercules, CA, United States); lysis buffer (Ambion, Austin, TX, United States); RNase-free yeast tRNA (Sigma-Aldrich Chemical Company, St Louis, MO, United States).

### Establishment of a CUMS Mouse Model With Depression-Like Behaviors

A total of 165 adult ICR male mice aged 8 weeks and weighing 19–23 g were purchased from the laboratory animal center of Jiangsu Province (Nanjing, Jiangsu, China) and reared under standard laboratory conditions. These mice were randomly housed in cages with a 12-h dark-light cycle, with lights on at 7:00 a.m., 60% humidity, air temperature of 24°C, and free access to water and food. All mice were acclimated for 1 week before CUMS treatment (Zhao L. et al., 2018; Guo et al., 2019). The 15 mice underwent control-operation were intragastrically administrated with DMSO. The remaining 150 mice were treated with 6 weeks of CUMS including 24-h fasting, 24-h water deprivation, 5-h physical restraint, 8-h of night lighting, 20-min horizontal oscillation, 24-h cage tilt at 45 °C, and 24-h environment of dirty cage (500 ml water and 250 g sawdust cushion). Among the CUMS-induced mice, 60 mice didn’t receive GP treatment (including 45 mice for adenovirus infection), 15 mice were intragastrically administrated with GP25 (25 mg/kg GP), 15 mice with GP50 (50 mg/kg GP) and 60 mice with GP100 (100 mg/kg GP, including 45 mice for adenovirus infection). The mice were intragastrically administrated 60 min before CUMS treatment at 10 mL/kg once a day. All the mice were weighed every 2 weeks (at the day 0, 14, 28, and 42 of CUMS induction). Six weeks after CUMS induction, behavioral tests were conducted to verify whether the CUMS mouse model was successfully established. The successfully modeled mice were deeply anesthetized by intraperitoneal injection with 3% pentobarbital sodium (P3761, Sigma-Aldrich Chemical Company, St Louis, MO, United States), followed by blood sample collection through orbital puncture, with isolation of the serum by centrifugation. After cervical dislocation, the brain was removed and the hippocampus tissues collected, frozen by immersion in liquid nitrogen and stored along with the plasma samples at −80°C.

### Behavioral Tests for the CUMS-Induced Depression-Like Behaviors

#### Sucrose Preference Test (SPT)

Twenty four after fasting and water deprivation, the mice were given a bottle of 1% sucrose water and a bottle of pure water. After 24 h, the SPT percentage was calculated by measuring the consumption of sucrose water and pure water as follows: SPT percentage (%) = (consumption of sucrose water/consumption of total liquid × 100%) (Leng et al., 2018).

#### Tail Suspension Test (TST)

Using the TST system (76-0780, Panlab, Barcelona, Spain), the mice were suspended on an acrylic rod with diameter of 15 cm and height of 30 cm for 6 min, and the video supervision tracking system (Smart 3.0, Panlab, Barcelona, Spain) was applied to measure the immobility time during the last 4 min of suspension (%).

#### Open Field Test (OFT)

A plastic box with size of 40 × 40 × 30 cm was equipped with the video supervision tracking system (Smart 3.0, Panlab, Barcelona, Spain) for behavioral tests in quiet surroundings. The mice were placed in the box for 10 min and the time spent in the central area (20 cm × 20 cm) was automatically recorded.

#### Forced Swimming Test (FST)

The FST system (760472, Panlab, Barcelona, Spain) along with a dielectric cylinder (20 cm diameter and 50 cm height) with pedestal was used for this test. Water temperature was 23–25°C, and the water depth was kept that the tip of mouse tail failed to touch the bottom of the container. On the first day, all mice were given 15 min pre-swimming training. On the next day, the video supervision tracking system (Smart 3.0, Panlab, Barcelona, Spain) was used to conduct 5 min FST for mice, with the immobility time of mice (%) recorded.

#### Morris Water Maze (MWM)

The water maze consisted of a circular water box (120 cm diameter) and a platform full of running water (22 ± 2°C), and the platform was placed 1–2 cm below the water surface. The mice were placed in one quadrant of the water maze and trained for five consecutive days to learn the platform position. With the camera installed above the water maze, the video supervision tracking system (Smart 3.0, Panlab, Barcelona, Spain) was used to record the swimming trail of mice. The time spent on test days to reach the platform (escape latency, with >120 s considered failure) was recorded. On day 6, the platform was removed, and the percentage of time mice spent in the target quadrant of the original platform was recorded.

### Culturing of Primary Neurons *in vitro*

The hippocampus tissues were placed in Ca^2+^- and Mg^2+^-free Hank’s balanced salt solution (HBSS) (14170112, Gibco, Carlsbad, CA, United States [the same as following corporation]) containing 1 mM sodium pyruvate and 10 mM HEPES, and then separated in the HBSS containing 0.125% trypsin (25200056) at 37°C for 10 min. Then, the cells were repeatedly triturated using a Pasteur pipette to split into single cells, and the DMEM containing 10% fetal bovine serum (FBS) was added for terminating the detachment. After 3-min, the supernatant was placed in a new centrifugation tube followed by another centrifugation at 2000 rpm for 2-min, and the Neurobasal medium containing B-27, 0.5 mM *L*-glutamine, 20 IU/ml penicillin and 20 IU/ml streptomycin were added in the pellet. Subsequently, the resuspended cells were seeded into 6-well plate coated by PDL (100 μg/ml) at the density of 4 × 10^6^ cells/well and cultured in the 5% CO_2_ incubator at 37°C, with half replacement of glutamic acid-free fresh medium every 2–3 days (Hu et al., 2012; Leon et al., 2016; Szychowski and Wojtowicz, 2016; Dang et al., 2018). After 3 days of culture, the purity of cultured neuronal (MAP2, green) and microglial (F4/80, red) cells was determined by immunofluorescence staining. The purity of the neurons used for experiment was about 95% (Leon et al., 2016).

### Cell Treatment

The CUMS-induced neurons were separately infected with the lentivirus of oe-NC, sh-NC, oe-Fezf1, sh-Fezf1, oe-Six3os1, inhibitor-NC, mimic-NC, miR-511-3p mimic and miR-511-3p inhibitor or in combination for 48 h. Other CUMS-induced neurons were firstly incubated with 10 μM GP for 24 h (Liu et al., 2017) and then separately infected with the lentivirus of sh-NC, sh-Fezf1, sh-Six3os1, mimic-NC, miR-511-3p mimic, miR-511-3p inhibitor, inhibitor-NC, oe-NC and oe-Fezf1 or in combination for 48 h. All lentiviruses were purchased from Shanghai Sangon Biotechnology Co. Ltd. (Shanghai, China), and the primer sequences and plasmids construction were conducted by Shanghai Sangon Biotechnology Co. Ltd. (Shanghai, China). Experiments were performed according to operation instructions.

### Dual-Luciferase Reporter Gene Assay

The target binding site between miR-511-3p and Fezf1 was predicted using an online analysis website^1^, and the site was predicted by another online analysis website^2^ between miR-511-3p and Six3os1. The 3’ untranslated region (3′UTR) sequences of Six3os1 and Fezf1 (Six3os1 wild type [Wt] and Fezf1 Wt) containing predicted binding sites were synthesized and introduced with mutant (Mut) sequences (Six3os1 Mut and Fezf1 Mut) into a pGL-3-basic vector (E1751, Promega, Madison, WI, United States). After digestion by restriction endonuclease, target fragments were inserted into pGL3 vector using T4 DNA ligase (M0204S, New England Biolabs, Beverly, MA, United States). The Renilla luciferase reporter plasmid and constructed firefly luciferase reporter plasmid were transfected into HEK293T cells by mimic-NC and miR-511-3p mimic, respectively. Cells were cultured in incubator with 5% CO_2_ under saturated humidity at 37°C, transfected for 48 h, collected and lysed. The luciferase activity was detected using Dual-Luciferase^®^ Reporter Assay System kit (E1910, Promega, Madison, WI, United States) on a GloMax^®^ 20/20 Luminometer detector (E5311, Promega, Madison, WI, United States), where the relative luciferase activity was calculated as the ratio of firefly luciferase activity to Renilla luciferase activity. All vectors were constructed by Shanghai Sangon Biotechnology Co. Ltd. (Shanghai, China).

### Hematoxylin Eosin (HE) Staining, Nissl Staining and TUNEL Staining

The brain was washed with phosphate buffered saline (PBS) at 4°C and fixed by immersion in 4% paraformaldehyde at 4°C. After dehydration in 20% sucrose, the brain was paraffin-embedded and cut into 10 μm-thick sections.

#### Hematoxylin Eosin Staining

Hippocampus tissue sections were selected, air-dried at room temperature, fixed for 30 s, stained with hematoxylin (at 60°C) for 60 s, differentiated by 1% hydrochloric ethanol and stained with eosin for 3 min. Subsequently, the sections were dehydrated in an ethanol series (70, 80, 95% and absolute ethanol; 5 min for each), cleared by xylene three times (5 min for each), and mounted by balsam. The changes of hippocampus structure were observed under a positive fluorescent microscope.

#### Nissl Staining

Complete hippocampus tissue sections were selected, air-dried under room temperature, fixed for 30 s, placed in cresyl violet acetate working liquid for 1-h without exposure to light, added into 70% ethanol, 80% ethanol, and 95% ethanol for color separation (about 10 s for each), and then added into color separation solution (absolute alcohol: chloroform: diethyl ether = 1: 1: 1) until clear color separation was observed. The sections were immersed in absolute alcohol twice (5-min each) and then permeabilized twice in xylene (4 min each), and mounted using balsam. The number of neurons was observed under positive fluorescent microscope (BX63, Olympus Optical Co., Ltd, Tokyo, Japan) (Guo et al., 2019).

TUNEL staining: with cell apoptosis detection kit (KHO1001, Thermo Fisher Scientific, MA, United States), the frozen sections were immersed in PBS, added into 200 mL citric acid buffer (0.1 mL, pH 6.0) heated at 90–95°C, irradiated by microwaves at 680 W (80% power) for 1 min, and immediately cooled by addition of 80 mL double distilled water (20–25°C). Then, the sections were added with 20% normal bovine serum at room temperature for 30 min, added with 50 μL TUNEL reaction mixture solution and incubated for 90 min at 37°C (NC without TUNEL reaction mixture solution). Subsequently, the sections were added with 3% H_2_O_2_ at room temperature for 10 min and incubated for 90 min at 37°C, then incubated with peroxisome (POD) (50 μL per section) for 30 min at 37°C, developed by diaminobenzidine (DAB)/H_2_O_2_, counterstained by hematoxylin, conventionally dehydrated, cleared and mounted with neutral balsam. The cells were observed and photographed under positive fluorescent microscope. The TUNEL positive cells showing deep brown staining of the nucleus were counted and calculated as the apoptotic cells.

### Fluorescence *in situ* Hybridization (FISH) Assay

The FISH kit (F32956, Thermo Fisher Scientific, MA, United States) was used to determine the location of Six3os1 in cells. Cells were incubated with digoxin-labeled Six3os1 probe (Sigma-Aldrich, SF, CA, United States), and stained with 4′,6-diamidino-2-phenylindole (DAPI) for 10 min. The confocal laser scanning microscope (FV1000, Olympus Optical Co., Ltd, Tokyo, Japan) was used to record the fluorescence image.

### Immunofluorescence Staining

Cells were inoculated into confocal cell culture dish for 24 h, fixed by 4% paraformaldehyde for 15 min. After being blocked with 5% goat serum (diluted to 0.3% in PBST) at room temperature for 1 h, the cells were incubated with block solution-diluted primary antibodies rat anti-mouse F4/80 (ab6640, 1:300) and rabbit anti-mouse MAP2 (ab32454, 1:300) at room temperature for 1 h. Then, the cells were incubated with red fluorescence protein (Cy3)-labeled secondary antibodies goat anti-rat (ab6953, 1: 500) and green fluorescence protein (FITC)-labeled goat anti-rabbit (ab6717, 1: 500) at room temperature for 1 h. Finally, the cells were mounted in a medium containing DAPI, air-dried and photographed. All antibodies above were purchased from Abcam (Cambridge, United Kingdom).

### Enzyme Linked Immunosorbent Assay (ELISA)

Enzyme linked immunosorbent assay kits were used to measure the mouse serum concentrations of tumor necrosis factor-α (TNF-α) (29-8321-65, Thermo Fisher Scientific, MA, United States), interleukin-1β (IL-1β) (29-8012-65, Thermo Fisher Scientific, MA, United States), IL-6 (29-8061-65, Thermo Fisher Scientific, MA, United States), superoxide dismutase (SOD) (DYC3419-2, R&D Systems, Minneapolis, MN, United States), malondialdehyde (MDA) (69-21068, Wuhan Msk Biotechnology Co., Ltd., Wuhan, China), glutathione (GSH) (69-80233, Wuhan Msk Biotechnology Co., Ltd., Wuhan, China) and catalase (CAT) (69-210385, Wuhan Msk Biotechnology Co., Ltd., Wuhan, China) (He et al., 2017). Experiments were conducted according to manufacturer’s instructions.

### Reverse Transcription Quantitative Polymerase Chain Reaction (RT-qPCR)

Total RNA was extracted using a Trizol kit, and then reversely transcribed into complementary DNA (cDNA) using TaqMan^TM^ MicroRNA Reverse Transcription Kit (for miRNA, 4366596, Thermo Fisher Scientific Inc., Waltham, MA, United States) and High-Capacity cDNA Reverse Transcription Kit (for mRNA, 4368813, Thermo Fisher Scientific Inc., Waltham, MA, United States). The RT-qPCR experiment was carried out according to the instructions of the RT-qPCR kit (11732020, Thermo Fisher Scientific Inc., Waltham, MA, United States). The primer sequences were designed and provided by Shanghai Sangon Biotechnology Co. Ltd. (Shanghai, China) (Table 1). With U6 as the internal reference for miR-511-3p and glyceraldehyde 3-phosphate dehydrogenase (GAPDH) as internal reference for Six3os1 and Fezf1, the fold changes of target genes between experimental group and control group were calculated by the 2^–ΔΔ*Ct*^ relative quantification method.

**TABLE 1:** Primer sequences for RT-qPCR.

Gene	Primer sequence (5′-3′)
Six3os1	F: TGTAGCAGCGGCGGATAAAT
	R: AGGCTTCCCAACAGGTTAGC
Fezf1	F: ACGCGACCACCAAAATGCTA
	R: TCGACGAGTTGAGATGCAGAG
GAPDH	F: AGGTCGGTGTGAACGGATTTG
	R: TGTAGACCATGTAGTTGAGGTCA
miR-511-3p	F: GCAGAATGTGTAGCAAAAGACA
	R: GGTCCAGTTTTTTTTTTTTTTTATCCT
U6	F: GCTTCGGCAGCACATATACTAAAAT
	R: CGCTTCACGAATTTGCGTGTCAT

*RT-qPCR, reverse transcription quantitative polymerase chain reaction; F, forward; R, reverse; GAPDH, glyceraldehyde 3-phosphate dehydrogenase; miR-511-3p, microRNA-511-3p.*

### Western Blot Analysis

The total protein was extracted from tissues or cells using a protein extraction kit (78501, Thermo Fisher Scientific, MA, United States), and the protein concentration was measured with the bicinchoninic acid assay kit (23229, Thermo Fisher Scientific, MA, United States). The concentration of protein was adjusted to 1 μg/μL, and the sample volume of each tube was set as 100 μL. The proteins were boiled at 100°C for denaturation and stored at −80°C for later analysis, followed by electrophoretic separation by 8–12% sodium dodecylsulphate (SDS) gel. After transfer onto a polyvinylidene fluoride (PVDF) membrane (1620177, Bio-Rad, Inc., Hercules, CA, United States), the samples were blocked with 5% skimmed milk or 5% bovine serum albumin (BSA) at room temperature for 1 h. Then the membrane was incubated with diluted monoclonal primary antibodies, namely GAPDH (ab181602, 1:5000), Fezf1 (orb29034, 1:1000), AKT (ab8805, 1:1000), phosphorylated (p)-AKT (ab81283, 1:1000), cleaved Caspase-3 (ab49822, 1:1000), Caspase-3 (ab13847, 1:1000), Bcl2-Associated X (Bax) (ab32503, 1:1000) and B-cell lymphoma-2 (Bcl-2) (ab692, 1:1000) respectively at 4°C overnight, followed by incubation with secondary antibodies horseradish peroxidase (HRP)-labeled goat anti-rabbit immunoglobulin G (IgG; ab6721, 1:5000) and rabbit anti-mouse IgG (ab6728, 1:5000) at room temperature for 1 h. All antibodies above were purchased from Abcam Inc. (Cambridge, United Kingdom) except Fezf1 (Biorbyt, Cambridge, United Kingdom). Subsequently, the membrane was immersed in ECL at room temperature for 1 min, and then exposed for image formation on the Image Quant LAS 4000C gel imager (General Electric Company, Boston, MA, United States). With GAPDH as internal reference, the relative expression of proteins was detected and expressed as the ratio of the gray values between the target band and internal reference band.

### RNA Immunoprecipitation (RIP) Assay

The RIP KIT (17-701, Millipore company, Billerica, MA, United States) was used to detect the binding between Six3os1 and AGO2 protein and between Fezf1 and AGO2 protein, with detection performed according to the manufacturer’s instructions. When the cell confluence in 6-well plate reached 80–90%, the medium was removed and the cells were added with 1 mL cold PBS and lysed with the same volume of RIPA Lysis Buffer (P0013B, Beyotime Institute of Biotechnology, Shanghai, China) on an ice bath, and centrifuged at 14,000 rpm for 10 min at 4°C to obtain supernatant. One part of the cell extracts was taken as input and the other part was taken to incubate with antibodies for co-precipitation. Specifically, 50 μL of magnetic beads from each co-precipitation reaction system were resuspended in 100 μL RIP Wash Buffer and incubated with 5 μg antibody for binding. The magnetic bead-antibody compound was resuspended in 900 μL RIP Wash Buffer and incubated with 100 μL cell extracts at 4°C overnight. Samples were placed on magnetic base to collect magnetic bead-protein compound. Then, samples and input were digested by protease K to extract RNA, which was used for subsequent detection of Six3os1 and Fezf1 expression. The antibodies used in the RIP assay were AGO2 (ab32381, 1:100, Abcam, Cambridge, United Kingdom) (mixed for 30 min at room temperature) and IgG (ab200699, 1:100, Abcam, Cambridge, United Kingdom) (used as NC).

### RNA Pull-Down Assay

Cells were transfected with biotin-labeled Bio-NC, Bio-Six3os1-Wt, Bio-Six3os1-Mut (50 nM for each), Bio-NC, Bio-Fezf1-Wt and Bio- Fezf1-Mut, respectively. After 48 h, the cells were collected and vortexed. Then, cells were incubated with cell lysis buffer for 10 min, and 50 mL sample cell lysates were sub-packed. The residual cell lysates were incubated with M-280 streptavidin magnetic bead pre-coated with RNase-free yeast tRNA at 4°C for 3 h, and followed by two washes with cold lysis solution, three washes with low salt buffer and one wash with high salt buffer. Finally, the bound RNA was purified by Trizol, and RT-qPCR was employed to detect the enrichment of miR-511-3p.

### Adenovirus Infection in Mice

The primer sequences and plasmids construction of sh-NC, sh-Fezf1, sh-Six3os1, oe-NC, oe-Fezf1, and oe-Six3os1 used for adenovirus construction (with green fluorescence) were completed by Shanghai Sangon Biotechnology Co. Ltd. (Shanghai, China), and experiment was conducted in accordance with instructions.

The CUMS-induced mice and CUMS-induced mice administered with GP100 used for adenovirus infection experiment. A total of 45 CUMS-induced mice were grouped by injecting with adenovirus of oe-NC + sh-NC, oe-Six3os1 + sh-NC and oe-Six3os1 + sh-Fezf1 (15 mice for each group). Another 45 CUMS-induced mice administered with GP100 were treated with injection of sh-NC + oe-NC, sh-Six3os1 + oe-NC and sh-Six3os1 + oe-Fezf1 (15 mice for each group). After anesthesia with 3% pentobarbital sodium, the mice were placed in stereotactic frame (SR-6M-HT, Felles Photonic Instruments, Shanghai, China). Using the Micro4 microinjection pump controller (15867, World Precision Instruments Inc., FL, United States), 1 μL adeno-associated virus (AAV) was injected into bilateral hippocampal regions (2.2 mm posterior to the bregma, 2.2 mm lateral to the midline, 1.8 mm dorsal to the bregma) at the rate of 300 nL/min. After injection, the incision was sutured and the mice were returned to their home cages for recovery. The behavioral tests were performed at the 10th day after intracerebral injection. Using a fluorescence microscope, hippocampus sections were observed whether green fluorescence expression existed, and the mice with green fluorescence expression were selected for subsequent biochemical analysis (Song et al., 2018; Han et al., 2019; Liang et al., 2019).

### RNA Sequencing and Bioinformatics Analysis

Sample collection: the brain tissues were collected from CUMS-induced mice and CUMS-induced mice with infection of GP100.

Construction of sequencing library: after extraction of total RNA, the rRNA in total RNA was removed using rRNA removal kit, and RNA was broken into the fragments with length of approximately 300 bp by means of ion interruption. With RNA used as template, 6 base random primer and reverse transcriptase sequences were synthesized into the first-strand cDNA, which was used as template to synthesize second-strand cDNA. After construction of the sequencing library, PCR amplification was applied for library fragment enrichment, and the library with size of 450 bp was selected. Subsequently, Agilent 2100 Bioanalyzer was used for library quality testing, followed by detection of total and effective concentrations in the library. Based on the effective concentration of library and the amount of data required from a library, the libraries containing different index sequences were mixed proportionally. Finally, the mixed libraries were uniformly diluted to 2 nM, and then formulated as a single-strand library through alkali denaturation.

Sequencing: after RNA extraction, purification and construction of sequencing library for samples, the libraries were treated with paired-end sequencing based on the Illumina HiSeq sequencing platform using the Next-Generation Sequencing (NGS).

Bioinformatics analysis: for the raw reads obtained from Illimina sequencing, the software cutadapt (v1.18) was first used to isolate the sequencing adaptor sequence in raw reads, and the internal software fqtools (v.0.1.6) was then used to filter out the low-quality sequences and to obtain clean reads, which served as the basis for the following analysis. Meanwhile, the Q30 value of clean reads was calculated. HiSAT2 (v.2.1.0) was employed to map the filtered clean reads to the mouse genome (*Mus musculus* GRCm38.90). The Deseq package in R software was used for data differential analysis with the screening threshold of | logFC| > 1 and FDR < 0.05. The starBse v2.0 database and RNA22 database were used to predict the downstream miRNAs of differentially expressed lncRNA Six3os1; meanwhile, miRDB database and TargetScan database were applied to predict the downstream target gene of miR-511-3p.

### Statistical Analysis

All data were processed by SPSS 21.0 statistical software (IBM Corp. Armonk, NY, United States). The measurement data conformed to normal distribution and homogeneity of variance were presented as mean ± standard deviation. Comparison of data between two groups was analyzed by independent sample test, while comparison of data among multiple groups was analyzed by one-way analysis of variance (ANOVA), and Bonferroni *post hoc* correction. Data at different time points among multiple groups were compared by repeated measures for ANOVA, and Bonferroni applied for *post hoc* test. *p* < 0.05 was considered as statistical significance.

## Results

### GP Alleviates the Depression-Like Behavior and Oxidative Stress of CUMS-Induced Mice

First, to explore whether GP affected depression-like behavior and oxidative stress of CUMS-induced mice, mice were administered with GP25, GP50 or GP100. Behavioral test results showed that, compared with control mice, the CUMS-induced mice exhibited significantly reduced sucrose preference, retention time in open field and memory ability, but obviously enhanced tail suspension time and forced swimming time (*p* < 0.05), which were rescued by administration of GP50 or GP100 (Figures 1A–E). No obvious difference was found in weight of mice with different treatments at the day 0 of CUMS induction (*p* > 0.05). At the day 14 of CUMS induction, compared with control mice, both the CUMS-induced mice and those administered with GP25 or GP50 showed significant weight loss (*p* < 0.05). At days 28 and 42, compared with control mice, CUMS-induced mice also showed obvious weight loss (*p* < 0.05), which was rescued by GP25 and GP50 (Figure 1F).

**FIGURE 1:** GP treatment relieves depression-like behavior and oxidative stress in CUMS-induced mice. The mice used for experiments were as follows: control mice, CUMS-induced mice and CUMS-induced mice administered with GP25, GP50, or GP100. **(A)** Sucrose preference of mice detected by SPT. **(B)** The retention time in open field of mice detected by OFT. **(C)** The immobility time of mice detected by TST. **(D)** The immobility time in water of mice detected by FST. **(E)** The percentage of time mice spent in the target quadrant of the platform detected by MWM. **(F)** the Weights of mice at the day 0, 14, 28, and 42 of CUMS induction. **(G)** The serum levels of TNF-α, IL-1β, and IL-6 in mice detected by ELISA. **(H)** The serum levels of SOD, MDA, GSH, and CAT in mice detected by ELISA. **(I)** The hippocampus tissues in mice observed by HE staining. **(J,K)** Representative views **(J)** and Nissl positive cell ratio **(K)** in hippocampus tissues of mice detected by Nissl staining. **(L,M)** Representative views **(L)** and apoptotic neuron ratio **(M)** in hippocampus tissues of mice detected by TUNEL staining. The measurement data were presented as mean ± standard deviation. Data comparison among multiple groups was analyzed by one-way ANOVA, followed by Tukey’s *post hoc* test. Data at different time points among multiple groups were compared by repeated measures ANOVA, and Bonferroni was applied for *post hoc* test. *n* = 15. *p < 0.05 *vs.* the CUMS-induced mice; #*p* < 0.05 *vs.* the control mice.

ELISA was conducted to detect the serum of TNF-α, IL-1β, IL-6, SOD, MDA, GSH, and CAT in mice. The results showed that compared with the control mice, the CUMS-induced mice presented a significant increase on serum levels of TNF-α, IL-1β, IL-6 and MDA, and serum levels of obvious reduction on SOD, GSH and CAT (*p* < 0.05); however, these results were abrogated by the GP25, GP50 or GP100 treatments (Figures 1G,H).

The HE staining showed that CUMS induction led to significant changes in hippocampus structure of mice with depression (Figure 1I). The ratio of Nissl positive cells was much lower in CUMS-induced mice than in control mice, which was rescued by GP100 treatment (*p* < 0.05; Figures 1J,K). TUNEL staining revealed that CUMS-induced mice exhibited significantly increased apoptotic neurons, which was rescued by GP100 treatment (Figures 1L,M). Thus, GP ameliorated the depression-like behavior and oxidative stress of CUMS-induced mice.

### GP Treatment Enhances Six3os1 Expression to Alleviate the Oxidative Stress of CUMS-Induced Neurons

The primary neurons were harvested from the hippocampus tissues of successfully modeled mice and cultured *in vitro* for 3 days, followed by morphology observation and immunofluorescence staining. The neuron had a purity of 95% (Figure 2A). After filtering out the low-quality sequences and cutting off the sequencing adaptor sequence in raw reads, the clean reads were obtained and mapped to mouse genome. We identified 55 differentially expressed genes (DEGs) including 49 mRNAs and 6 lncRNAs (Figure 2B). Among these DEGs, Six3os1 showed significantly increased expression in mice with GP treatment (Figure 2C). Further, RT-qPCR was employed to examine the Six3os1 expression in mouse models and neurons. The results revealed significantly lower Six3os1 expression in CUMS-induced mice than control mice (Supplementary Figure S2A). On the contrary, significantly higher Six3os1 expression was observed in CUMS-induced mice administered with GP50 or GP100 than in CUMS-induced mice, and obviously higher expression of Six3os1 was also found in CUMS-induced neurons treated with GP, which was much higher than that in CUMS-induced neurons (*p* < 0.05; Figure 2D). Then, Six3os1 was overexpressed in CUMS-induced neurons, and was knocked down in CUMS-induced neurons treated with GP. RT-qPCR documented that Six3os1 expression was obviously increased after oe-Six3os1 treatment in CUMS-induced neurons, and significantly decreased after sh-Six3os1 treatment in CUMS-induced neurons treated with GP (Figure 2E). Then, ELISA was employed to measure the contents of SOD, GSH, CAT, and MDA in neurons. In CUMS-induced neurons, oe-Six3os1 treatment led to profoundly elevated contents of SOD, GSH and CAT but markedly lowered MDA content; however, the result was opposite after sh-Six3os1 treatment in CUMS-induced neurons treated with GP (Figure 2F).

**FIGURE 2:** GP treatment ameliorated the oxidative stress of CUMS-induced neurons through upregulation of Six3os1. **(A)** The morphology of the neurons *in vitro* and purity of neurons detected by immunofluorescence staining. **(B)** The heatmap of predicted DEGs, with abscissa representing logFC value and ordinate representing –log_10_ *p*-value; each pot in the figure represents one gene, with red pot representing the highly expressed gene in cells with GP treatment and green pot representing the poorly expressed gene in cells with GP treatment. **(C)** The Six3os1 expression detected by RNA-seq data analysis, with a green boxplot representing control cells and red boxplot representing cells with GP treatment; the values at upper right are corrected *p*-values. **(D)** Six3os1 expression in mice (*n* = 15) and neurons after CUMS and GP treatment examined by RT-qPCR. **(E)** Six3os1 expression in cells after treatments of sh-Six3os1 and oe-Six3os1 determined by RT-qPCR. **(F)** The contents of SOD, GSH, CAT, and MDA in neurons after treatments of sh-Six3os1 and oe-Six3os1 detected by ELISA. **(G–K)** Immunoblots **(G)** and quantitation of Bax **(H)**, Cleaved caspase-3 **(I)**, Bcl-2 **(J)**, and caspase-3 **(K)** protein expression normalized to GAPDH in neurons after treatments with sh-Six3os1 and oe-Six3os1 examined by Western blot analysis. The measurement data were presented as mean ± standard deviation. Data between two groups were compared by independent sample *t*-test, and data among multiple groups were analyzed by one-way ANOVA, followed by Tukey’s *post hoc* test. Cell experiments were repeated three times. *p < 0.05 *vs.* CUMS-induced mice, CUMS-induced neurons, oe-NC treatment or sh-NC treatment.

Further, the effect of Six3os1 on neuronal apoptosis was assessed by Western blot analysis. As depicted in Figures 2G–K, in CUMS-induced neurons, oe-Six3os1 treatment significantly reduced Bax and cleaved-caspase3 expression and remarkably elevated Bcl-2 expression. Nevertheless, the result was opposite after treating with sh-Six3os1 in CUMS-induced neurons (before GP treatment). However, caspase-3 expression did not change in cells with any treatment (*p* > 0.05). Thus, GP treatment upregulated Six3os1 expression and alleviated the oxidative stress of CUMS-induced neurons.

### Six3os1 Alleviates Oxidative Stress in CUMS-Induced Neurons Through Inhibiting miR-511-3p

The findings above revealed increased Six3os1 expression in CUMS-induced mice upon GP treatment, and the binding site between Six3os1 and miR-511-3p was found through the Star Base (Figure 3A). FISH showed that Six3os1 was expressed both in cytoplasm and nucleus (Figure 3B). RT-qPCR showed that miR-511-3p expression was upregulated in CUMS-induced mice (Supplementary Figure S2A), and versus CUMS-induced mice, CUMS-induced mice administered with GP50 or GP100 had decreased miR-511-3p expression. miR-511-3p expression was significantly decreased in CUMS-induced neurons treated with GP, compared with CUMS-induced neurons (*p* < 0.05; Figure 3C). To further determine the targeting relationship between Six3os1 and miR-511-3p, the dual-luciferase reporter gene assay was employed. The results revealed that miR-511-3p mimic treatment significantly suppressed the luciferase activity in Six3os1-Wt (*p* < 0.05) but had no obvious effect on the luciferase activity in Six3os1-Mut (*p* > 0.05; Figure 3D). The RIP assay displayed that the enrichment of miR-511-3p and Six3os1 was significantly higher in AGO2 than in IgG (*p* < 0.05; Figure 3E). The results of RNA pull-down showed that miR-511-3p expression was markedly increased after treatment of Bio-Six3os1-Wt (Figure 3F). All the results support a targeting relationship between miR-511-3p and Six3os1.

**FIGURE 3:** Six3os1 alleviates oxidative stress in CUMS-induced neurons through inhibiting miR-511-3p. **(A)** The targeting relationship between Six3os1 and miR-511-3p predicted by StarBase website. **(B)** The subcellular localization of Six3os1. **(C)** miR-511-3p expression in mice (*n* = 15) and neurons after CUMS and GP treatment detected by RT-qPCR. **(D)** The targeting relationship between Six3os1 and miR-511-3p verified by dual-luciferase reporter gene assay. **(E)** The targeting relationship between Six3os1 and miR-511-3p determined by RIP assay. **(F)** The targeting relationship between Six3os1 and miR-511-3p determined by RNA pull down. **(G)** miR-511-3p expression in neurons after treatment of miR-511-3p inhibitor and miR-511-3p mimic detected by RT-qPCR. **(H)** SOD, GSH, CAT, and MDA contents in neurons after alteration of Six3os1 and miR-511-3p examined by ELISA. **(I–L)** Quantitation of Bax **(I)**, Cleaved caspase-3 **(J)**, Bcl-2 **(K)**, and caspase-3 **(L)** protein expression normalized to GAPDH in cells after alteration of Six3os1 and miR-511-3p detected by Western blot analysis. The measurement data were presented as mean ± standard deviation. Data between two groups were compared by independent sample *t*-test, and data among multiple groups were analyzed by one-way ANOVA, followed by Tukey’s *post hoc* test. Cell experiments were repeated three times. ^∗^*p* < 0.05 *vs.* CUMS-induced mice, CUMS-induced neurons, inhibitor-NC + sh-NC, mimic-NC + oe-NC, oe-NC or sh-NC. ^#^*p* < 0.05 *vs.* miR-511-3p inhibitor + sh-NC or miR-511-3p mimic + oe-NC.

We next investigated whether miR-511-3p augmented the oxidative stress of neurons in mice with CUMS-induced depression. First, RT-qPCR showed that miR-511-3p expression progressively decreased after miR-511-3p inhibitor treatment in the CUMS-induced neurons, and significantly increased after miR-511-3p mimic treatment in the GP-treated CUMS-induced neurons (Figure 3G). Subsequently, CUMS-induced neurons were treated with inhibitor-NC + sh-NC, miR-511-3p inhibitor + sh-NC or miR-511-3p inhibitor + sh-Six3os1. CUMS-induced neurons treated with GP were infected with the lentivirus of mimic-NC + oe-NC, miR-511-3p mimic + oe-NC or miR-511-3p mimic + oe-Six3os1. ELISA revealed that in the CUMS-induced neurons, the miR-511-3p inhibitor treatment led to significantly increased contents of SOD, GSH, and CAT but a remarkable decrease in MDA content; these effects were abolished by sh-Six3os1 treatment. Besides, in the CUMS-induced neurons treated with GP, reduced SOD, GSH and CAT and increased MDA content were found after treatment of miR-511-3p mimic, which was negated by oe-Six3os1 treatment (Figure 3H). According to results from Western blot analysis, in the CUMS-induced neurons, miR-511-3p inhibitor significantly reduced Bax and cleaved-caspase3 expression but induced Bcl-2 expression, which was abrogated by sh-Six3os1 treatment. Also, in the CUMS-induced neurons treated with GP, Bax and cleaved-caspase3 expression was markedly enhanced but Bcl-2 expression was significantly reduced by miR-511-3p mimic (negated by oe-Six3os1). The expression of caspase-3 showed no pronounced difference in cells with any treatment (*p* > 0.05; Figures 3I–L). Therefore, miR-511-3p augmented the oxidative stress of CUMS-induced neurons, while Six3os1 suppressed the effect of miR-511-3p.

### Six3os1 Elevates Fezf1 Expression Through Inhibition of miR-511-3p

The above findings revealed that miR-511-3p was highly expressed in mice with depression and induced oxidative stress in CUMS-induced neurons. To further explore the downstream regulatory mechanism of miR-511-3p, miRDB and TargetScan databases were employed to predict the downstream target genes of miR-511-3p. Upon interesting the predicted genes, 564 potential downstream target genes were obtained (Figure 4A). Through differential analysis, two downstream target genes (Prkch and Fezf1) were found to be differentially expressed (Figure 4B). Fezf1 expression in CUMS-induced mice treated with GP100 (13.60234) was 40-fold higher than that in CUMS-induced mice (0.33) (Figures 4B,C). The online prediction website TargetScan revealed the binding site between Fezf1 and miR-511-3p (Figure 4D). Further, Western blot analysis revealed lower Fezf1 protein expression in CUMS-induced mice than control mice (Supplementary Figure S2B). RT-qPCR and Western blot analysis showed that, compared with CUMS-induced mice, CUMS-induced mice treated with GP50 and GP100 exhibited significantly increased Fezf1 expression (*p* < 0.05). In comparison with CUMS-induced neurons, elevated Fezf1 expression was observed in CUMS-induced neurons with GP treatment (*p* < 0.05; Figures 4E–G). The results of dual-luciferase reporter gene assay revealed that miR-511-3p mimic markedly suppressed the luciferase activity of Fezf1-Wt (*p* < 0.05) but did not affect the luciferase activity of Fezf1-Mut (*p* > 0.05; Figure 4H). These findings led to a conclusion that miR-511-3p targeted Fezf1.

**FIGURE 4:** Six3os1 binds to miR-511-3p and upregulates Fezf1. **(A)** The downstream target genes of miR-511-3p predicted by the TargetScan and miRDB databases; two circles in the figure represent the predicted results of the TargetScan and miRDB databases, with the central part representing the intersection of the predicted results. **(B)** Intersection of the predicted target genes of miR-511-3p and differentially expressed genes, with the central part representing their intersection. **(C)** Fezf1 expression detected by RNA-seq data detection, with green boxplot representing CUMS induction and red boxplot representing CUMS induction with GP treatment. The values at upper right were corrected *p*-values. **(D)** The targeting relationship between Fezf1 and miR-511-3p predicted by the TargetScan website. **(E)** Fezf1 mRNA expression in mice (*n* = 15) and neurons after CUMS and GP treatment detected by RT-qPCR. **(F,G)** Immunoblots **(F)** and quantitation of Fezf1 **(G)** protein expression normalized to GAPDH in mice (*n* = 15) and neurons after CUMS and GP treatment examined by Western blot analysis. **(H)** The targeting relationship between Fezf1 and miR-511-3p verified by dual-luciferase reporter gene assay. **(I)** Fezf1 mRNA expression in CUMS-induced neurons after alteration of Six3os1 and miR-511-3p detected by RT-qPCR. **(J)** Fezf1 mRNA expression in CUMS-induced neurons with GP treatment neurons after alteration of Six3os1 and miR-511-3p detected by RT-qPCR. **(K–M)** Immunoblots **(K)** and quantitation **(L,M)** of Fezf1 protein expression normalized to GAPDH in CUMS-induced neurons after alteration of Six3os1 and miR-511-3p determined by Western blot analysis. The measurement data were presented as mean ± standard deviation. Data between two groups were compared by independent sample *t-*test, and data among multiple groups were analyzed by one-way ANOVA, followed by Tukey’s *post hoc* test. Cell experiment was repeated three times. *p < 0.05 *vs.* CUMS-induced mice, CUMS-induced neurons, oe-NC + mimic-NC, sh-NC + inhibitor-NC, mimic-NC or inhibitor-NC; ^#^*p* < 0.05 *vs.* oe-Six3os1 + mimic-NC or sh-Six3os1 + inhibitor-NC.

Subsequently, we investigated whether Six3os1 elevated Fezf1 expression through regulation of miR-511-3p. Therefore, CUMS-induced neurons were treated with oe-NC + mimic-NC, oe-Six3os1 + mimic-NC, inhibitor-NC, miR-511-3p inhibitor or oe-Six3os1 + miR-511-3p mimic. CUMS-induced neurons treated with GP were infected with the lentivirus of sh-NC + inhibitor-NC, sh-Six3os1 + inhibitor-NC, mimic-NC, miR-511-3p mimic or sh-Six3os1 + miR-511-3p inhibitor. As documented by RT-qPCR and Western blot analysis (Figures 4I–M), in CUMS-induced neurons, oe-Six3os1 treatment contributed to obviously increased Fezf1 expression, which was reversed by miR-511-3p mimic treatment. However, miR-511-3p inhibitor treatment also induced increase in Fezf1 expression. In CUMS-induced neurons with GP treatment, Fezf1 expression was significantly reduced after silencing Six3os1, which was abrogated by miR-511-3p inhibitor. The reduced Fezf1 expression was also found after miR-511-3p mimic treatment. In conclusion, Six3os1 enhanced Fezf1 expression by binding to miR-511-3p.

### Six3os1 Alleviates Oxidative Stress of CUMS-Induced Neurons Through Activation of Fezf1/AKT Axis by Binding to miR-511-3p

The aforementioned findings suggested that Six3os1 elevated Fezf1 expression by binding to miR-511-3p. We then probed whether Fezf1 could alleviate the oxidative stress of CUMS-induced neurons. Fezf1 was overexpressed or knocked down in CUMS-induced neurons, followed by RT-qPCR and Western blot analysis. As demonstrated in Figures 5A–C, oe-Fezf1 treatment significantly increased Fezf1 expression in CUMS-induced cells, while sh-Fezf1 treatment progressively decreased Fezf1 expression in CUMS-induced cells with GP treatment.

**FIGURE 5:** Six3os1 activates the Fezf1/AKT axis by binding to miR-511-3p, thus ameliorating oxidative stress of CUMS-induced neurons. **(A)** Fezf1 mRNA expression in neurons after alteration of Fezf1 detected by RT-qPCR. **(B,C)** Immunoblots **(B)** and quantitation **(C)** of Fezf1 protein expression normalized to GAPDH in neurons after alteration of Fezf1 examined by Western blot analysis. The CUMS-induced neurons were treated with oe-NC + sh-NC, oe-Fezf1 + sh-NC, oe-Six3os1 + sh-Fezf1, miR-511-3p inhibitor + sh-Fezf1, oe-Six3os1 + sh-NC or miR-511-3p inhibitor + sh-NC, and CUMS-induced neurons with GP treatment were infected with oe-NC + sh-NC, oe-NC + sh-Fezf1, oe-NC + sh-Six3os1, oe-Fezf1 + sh-Six3os1, miR-511-3p mimic + oe-NC or miR-511-3p mimic + oe-Fezf1. **(D–G)** SOD **(D)**, GSH **(E)**, CAT **(F),** and MDA **(G)** contents in neurons determined by ELISA. **(H–K)** Quantitation of Bax **(H)**, Cleaved-caspase3 **(I)**, Bcl-2 **(J),** and caspase3 **(K)** protein expression normalized to GAPDH in neurons detected by Western blot analysis. **(L–N)** Immunoblots **(L)** and quantitation of AKT expression **(M)** and p-AKT **(N)** normalized to GAPDH in neurons determined by Western blot analysis. The measurement data were presented as mean ± standard deviation. Data between two groups were compared by independent sample *t-*test, and data among multiple groups were analyzed by one-way ANOVA, followed by Tukey’s *post hoc* test. Cell experiments were repeated three times. ^∗^*p* < 0.05 *vs.* oe-NC + sh-NC, oe-Six3os1 + sh-NC, miR-511-3p inhibitor + sh-NC, oe-NC + sh-Six3os1 or miR-511-3p mimic + oe-NC.

Further, ELISA was used to detect the expression of oxidative stress-related factors. In CUMS-induced neurons, Fezf1 overexpression triggered significantly increased SOD, GSH and CAT contents but significantly decreased MDA content, whereas opposite results were seen after treatment of oe-Six3os1 + sh-Fezf1 or miR-511-3p inhibitor + sh-Fezf1 in comparison with the effect of oe-Six3os1 + sh-NC or miR-511-3p inhibitor + sh-NC treatments, respectively (*p* < 0.05). In CUMS-induced neurons with GP treatment, SOD, GSH, and CAT contents were diminished but the MDA content was profoundly increased by silencing Fezf1. In comparison with treatment of oe-NC + sh-Six3os1 or miR-511-3p mimic + oe-NC respectively, treatment with oe-Fezf1 + sh-Six3os1 or miR-511-3p mimic + oe-Fezf1 induced obviously increased SOD, GSH, and CAT contents but significantly reduced MDA content (*p* < 0.05; Figures 5D–G).

We then clarified the effect of Fezf1 on neuronal apoptosis using Western blot analysis. As displayed in Figures 5H–K, in CUMS-induced cells, Bax and Cleaved caspase-3 expression was reduced but Bcl-2 expression enhanced after overexpression of Fezf1 (*p* < 0.05). In comparison with oe-Six3os1 + sh-NC treatment, oe-Six3os1 + sh-Fezf1 treatment significantly increased Bax and Cleaved caspase-3 expression but obviously decreased Bcl-2 expression (*p* < 0.05). Significant enhancement Bax and Cleaved caspase-3 expression and marked reduction of Bcl-2 expression were found after treatment of miR-511-3p inhibitor + sh-Fezf1 relative to treatment of miR-511-3p inhibitor + sh-NC (*p* < 0.05). In CUMS-induced cells with GP treatment, silence of Fezf1 significantly elevated Bax and Cleaved caspase-3 expression but reduced Bcl-2 expression. These effects were reversed after treatment of oe-Six3os1 + sh-Fezf1 or miR-511-3p inhibitor + sh-Fezf1 in contrast to the treatment of oe-Six3os1 + sh-NC or miR-511-3p inhibitor + sh-NC respectively (*p* < 0.05). Additionally, the expression of Caspase-3 was unaffected in cells by any treatment (*p* > 0.05).

Then Western blot analysis was performed to investigate the correlation between Fezf1 and AKT signaling pathway. This showed that the extent of AKT phosphorylation was decreased in CUMS-induced mice relative to control mice (Supplementary Figure S2B). In CUMS-induced neurons, the co-treatment with oe-Fezf1 and sh-NC led to significantly increased AKT phosphorylation, relative to treatment of oe-NC + sh-NC, but phosphorylation was reduced following treatment with oe-Six3os1 + sh-Fezf1 or miR-511-3p inhibitor + sh-Fezf1, compared to the treatment with oe-Six3os1 + sh-NC or miR-511-3p inhibitor + sh-NC respectively (*p* < 0.05). After Fezf1 was knocked down in CUMS-induced neurons with GP treatment, we observed reduced AKT phosphorylation. In comparison with oe-NC + sh-Six3os1 treatment, oe-Fezf1 + sh-Six3os1 treatment significantly increased AKT phosphorylation (*p* < 0.05). Compared with miR-511-3p mimic + oe-NC treatment, miR-511-3p mimic + oe-Fezf1 treatment also enhanced AKT phosphorylation (*p* < 0.05). There was no obvious difference in AKT expression in neurons with different treatments (*p* > 0.05; Figures 5L–N). These findings suggested that Six3os1 enhanced Fezf1 expression by binding to miR-511-3p, and that Fezf1 activated AKT signaling pathway to alleviate the oxidative stress of CUMS-induced neurons.

### Six3os1 Overexpression Ameliorates Oxidative Stress in CUMS-Induced Mice *in vivo* by Upregulating Fezf1

Subsequently, we clarified the effects of Six3os1 and Fezf1 in mice *in vivo*. First, the adenovirus was injected into the hippocampal regions of mice to detect the changes of depression-like behavior, which revealed the expression of green fluorescence in the hippocampus tissue sections (Figure 6A). Then, RT-qPCR was employed to detect the adenovirus infection efficiency (Figure 6B). In CUMS-induced mice, compared with oe-NC + sh-NC treatment, oe-Six3os1 + sh-NC treatment resulted in significantly increased Six3os1 and Fezf1 expression (*p* < 0.05). On the other hand, oe-Six3os1 + sh-Fezf1 treatment induced significantly increased Six3os1 expression but progressively decreased Fezf1 expression relative to effects of Six3os1 + sh-NC (*p* < 0.05). In CUMS-induced mice administered with GP, sh-Six3os1 + oe-NC treatment presented with remarkable reduction of Six3os1 and Fezf1 expression compared to sh-NC + oe-NC treatment (*p* < 0.05). Conversely, sh-Six3os1 + oe-Fezf1 treatment led to significantly diminished Six3os1 expression but elevated Fezf1 expression relative to sh-Six3os1 + oe-NC treatment (*p* < 0.05). Western blot analysis revealed that in CUMS-induced mice, Fezf1 expression was markedly increased after oe-Six3os1 + sh-NC treatment but significantly reduced by Six3os1 + sh-Fezf1 treatment relative to treatment of oe-NC + sh-NC (*p* < 0.05). In CUMS-induced mice with GP treatment, Fezf1 showed diminished expression following sh-Six3os1 + oe-NC treatment, but was significantly upregulated by sh-Six3os1 + oe-Fezf1 treatment in comparison with sh-NC + oe-NC treatment (*p* < 0.05; Figures 6C,D).

**FIGURE 6:** Overexpressed Six3os1 greatly alleviates oxidative stress of neurons in mice with CUMS-induced depression *in vivo*. CUMS-induced mice were injected with adenovirus of oe-NC + sh-NC, oe-Six3os1 + sh-NC and oe-Six3os1 + sh-Fezf1, and CUMS-induced mice administered with GP100 were injected with sh-NC + oe-NC, sh-Six3os1 + oe-NC and sh-Six3os1 + oe-Fezf1. **(A)** The injection of adenovirus and green fluorescence expression. **(B)** Six3os1 and Fezf1 expression in mice detected by RT-qPCR. **(C,D)** Immunoblots **(C)** and quantitation **(D)** of Fezf1 protein expression normalized to GAPDH in mice examined by Western blot analysis. **(E)** Sucrose preference (%) of mice after different treatments. **(F)** Retention time in open field (s) of mice after different treatments. **(G)** Memory ability of mice after different treatments evaluated by Morris water maze. **(H)** Tail suspension time (s) of mice after different treatments. **(I)** Forced swimming time (s) of mice after different treatments. **(J)** The weight of mice at day 42. **(K)** SOD, GSH, CAT, and MAD contents in mice determined by ELISA. The measurement data were presented as mean ± standard deviation. Data between two groups were compared by independent sample *t-*test, and data among multiple groups were analyzed by one-way ANOVA, followed by Tukey’s *post hoc* test. *p < 0.05 *vs.* CUMS-induced mice treated with oe-NC + sh-NC and the CUMS-induced mice administered with GP after treatment of sh-NC + oe-NC; ^#^*p* < 0.05 *vs.* the CUMS-induced mice treated with oe-Six3os1 + sh-NC and CUMS-induced mice administered with GP after treatment of sh-Six3os1 + oe-NC.

The results of behavioral tests revealed that in CUMS-induced mice, the sucrose preference, retention time in open field and memory ability were significantly enhanced while the tail suspension time and forced swimming time drastically reduced after overexpression of Six3os1, which was abrogated by sh-Fezf1. In CUMS-induced mice with GP treatment, there was marked decrease of sucrose preference, retention time in open field and memory ability and increased tail suspension time and forced swimming time after silencing Six3os1, which was abolished by overexpressing Fezf1 (Figures 6E–I). Additionally, in CUMS-induced mice, Six3os1 overexpression contributed to obviously increased weight gain of mice, which was negated with sh-Fezf1 treatment. In CUMS-induced mice with GP treatment, the Six3os1-downregulated mice exhibited significantly lowered weight, which was normalized following ectopic expression of Fezf1 (Figure 6J). To sum up, Six3os1 and Fezf1 significantly alleviated the depression-like behavior of CUMS-induced mice.

ELISA analysis in CUMS-induced mice showed reduced contents of SOD, GSH, and CAT but MDA content was increased after overexpressing Six3os1, which was reversed by Fezf1 silencing. In CUMS-induced mice with GP treatment, SOD, GSH and CAT contents declined but MDA content increased in Six3os1-downregulated mice, which was abolished by upregulating Fezf1 (Figure 6K). In summary, overexpression of Six3os1 alleviated oxidative stress of CUMS-induced mice via Fezf1 upregulation.

## Discussion

Depression, a major burden around the world, brings serious disability, now ranking in second place with respect to adjusted life years of disability among all age groups (Planchez et al., 2019). Previous studies have shown obvious damage and hippocampal neuron loss in depression model rat hippocampus (Bakhtiarzadeh et al., 2018; Zhao L. et al., 2018). The results we obtained also showed consistent changes, whereas the GP treatment could alleviate CUMS-induced depression-like behavior and hippocampal damage in mice. Evidence exists reporting that GP treatment confers protective effects against depression (Wang et al., 2016). Additionally, Six3os1 exerted effects on neuronal and oligodendrocyte differentiation (Ramos et al., 2013). Accordingly, we hypothesized significant roles of GP and Six3os1 in the mice with depression-like behavior induced by CUMS. Through a series of experiments, the present study eventually illustrated that GP upregulated Six3os1 expression, which then alleviated the oxidative stress in mice with CUMS-induced depression-like behavior through activation of the miR-511-3p-mediated Fezf1/AKT signaling pathway.

We conducted behavioral tests and oxidative stress analysis on CUMS-induced mice, and obtained experimental data consistent with the hypothesis, which is also consistent with the findings of Zhao Y. et al. (2018). First, we found that miR-511-3p was highly expressed but Six3os1 and Fezf1 were downregulated in mice with CUMS-induced depression-like behavior and these changes promoted the oxidative stress of mice with CUMS-induced depression-like behavior. This finding supports earlier results that miR-511 is highly expressed in the prefrontal cortex of CUMS-induced adolescent rats (Xu et al., 2019). In addition, highly expressed miR-511 was observed in neural progenitor cells from depressed human subjects (Maheu et al., 2015). Importantly, miR-511 enhanced neuronal differentiation in cells to induce the development of primary neurons in culture (Zheng et al., 2016). More importantly, miR-511-3p expression was decreased but Six3os1 and Fezf1 expression was elevated in CUMS-treated mice following GP treatment. Fezf1 was reported to be an essential factor in sensory neuron identity and olfactory development (Eckler et al., 2011), and can mediate the development of human neurons (Liu et al., 2018). In fact, Wang et al. (2019) have shown alterations in small non-coding RNA networks and coding genes in the brain of human and animal depression models, suggesting that lncRNA-linked complex trait-specific crosstalk may play a vital role in the progression of depression.

Besides, Six3os1 was suggested to elevate Fezf1 expression by binding to miR-511-3p to alleviate depression symptoms in the CUMS model. GP-induced Six3os1 overexpression suppressed the oxidative stress and neuronal apoptosis of CUMS-induced mice by enhancing Fezf1-dependent AKT signaling pathway via miR-511-3p inhibition. Specifically, in CUMS-induced mice, the contents of SOD, GSH, and CAT were diminished and MDA content was elevated in response to Six3os1 overexpression, which was reversed by Fezf1 knockdown. However, knockdown of Six3os1 reduced the SOD, GSH, and CAT contents and elevated MDA content in CUMS-induced mice with GP treatment, which was negated by upregulating Fezf1. In other studies, GP treatment alleviated depression-like behavior caused by repeated restraint stress through suppression of neuronal apoptosis via the modulation of the GLP-1R/AKT signaling pathway (Zhao L. et al., 2018). Moreover, GP can correct depression-like behavior of offspring from prenatally stressed mice by repressing DNA methyltransferase 1, i.e., an epigenetic mechanism (Zhao L. et al., 2018). GP treatment alleviated the cisplatin-induced renal tissue damage by abrogating oxidative stress and disrupting cell death pathways, hence improving renal function (Mahgoub et al., 2017). Moreover, loss of Fezf1 blocks neural differentiation of human embryonic stem cells and abrogates the pluripotency exit of human embryonic stem cells in neural specification (Liu et al., 2018). Also, overexpressed Fezf1 reportedly attenuated glioma cell apoptosis through activation of the AKT signaling pathway (Yu et al., 2017, 2018). Activation of the AKT signaling pathway stimulated by baicalin suppressed the CUMS-induced inflammation (Yu et al., 2017). Mechanistically, our present results further revealed that up-regulating Six3os1 could reduce the oxidative stress of neurons in CUMS-induced mice, and that Six3os1 elevated Fezf1 expression through competitively binding to miR-511-3p. Although the mechanism by which GP treatment induced changes in the expression of Six3os1 and miR-511-3p to alleviate depression-like behavior is not clear, we speculate that GP may induce subsequent changes through the induction of epigenetic changes such as DNA methylation, but the specific mechanism remains to be further explored.

Taken together, the key findings obtained from this study suggested the potential effect of GP treatment on restricting oxidative stress of CUMS-induced mice with depression-like behavior by upregulating Six3os1 through regulation of miR-511-3p-dependent Fezf1/AKT axis (Figure 7). The functional mechanism of GP-mediated Six3os1 *via* miR-511-3p/Fezf1/AKT unveiled in present study provided novel therapeutic hints for depression prevention and treatment. Nevertheless, it should also be noted whether the therapeutic target is applicable to human beings requires to be further verified. Additional studies have also suggested to compare the binding efficiency of miR-511-3p on Six3os1 and Fezf1 mRNA in order to further confirm that Six3os1 regulates Fezf1 expression by disrupting the binding of miR-511-3p on mRNA of Fezf1. Moreover, the findings provided in this study are preliminary, indicating more studies in this area are required in the future.

**FIGURE 7:** The molecular mechanism of GP treatment mediating oxidative stress in mice with depression-like behavior *via* the Six3os1/Fezf1/AKT. In CUMS-induced mice, miR-511-3p targets and inhibits Fezf1, thus stimulating oxidative stress of neurons. After GP treatment, Six3os1 expression is upregulated, which increases Fezf1 expression by binding to miR-511-3p and then activates AKT signaling pathway, thus alleviating oxidative stress in mice with depression-like behavior.

## Data Availability Statement

The raw data supporting the conclusions of this article will be made available by the authors, without undue reservation, to any qualified researcher.

## Ethics Statement

The animal use and experimental procedures in this study were conducted in accordance with the Guide for the Care and Use of Laboratory Animals published by the National Institutes of Health. The animal experiments were approved by the animal ethics committee of Heilongjiang Academy of Chinese Medical Sciences.

## Author Contributions

TZ, JZ, YZ, YL, KS, HL, YJ, and JW designed the study. GD, CM, TZ, JZ, and YZ collated the data, carried out the data analyses, and produced the initial draft of the manuscript. YL, KS, and HL contributed to drafting the manuscript. All authors have read and approved the final submitted manuscript.

## Conflict of Interest

The authors declare that the research was conducted in the absence of any commercial or financial relationships that could be construed as a potential conflict of interest.

## Footnotes

1 http://www.targetscan.org/

2 http://starbase.sysu.edu.cn/index.php

## Supplementary Material

FIGURE S1 Structure of geniposide from *Gardenia jasminoides* Ellis fruits.

FIGURE S2 High miR-511-3p expression and poor expression of Six3os1 and Fezf1 in CUMS-induced mice. **(A)** Six3os1 and miR-511-3p expression in mice measured by RT-qPCR. **(B)** Immunoblots (left) and quantitation (right) of Fezf1 and AKT protein expression normalized to GAPDH in mice examined by Western blot analysis. Data between two groups were compared by independent sample *t-*test. Cell experiments were repeated three times. ^∗^*p* < 0.05 *vs.* control mice.

## Abbreviations

Bax: Bcl2-Associated X
CAT: catalase
CUMS: chronic unpredictable mild stress
DMEM: Dulbecco’s modified eagle medium
ELISA: enzyme linked immunosorbent assay
FISH: fluorescence in situ hybridization
FST: forced swimming test
GLP-1R: glucagon-like peptide-1 receptor
GP: geniposide
GSH: glutathione
HBSS: Hank’s balanced salt solution
HE: hematoxylin eosin
MDA: malondialdehyde
MWM: Morris water maze
OFT: open field test
RIP: RNA immunoprecipitation
RT-qPCR: reverse transcription quantitative polymerase chain reaction
SOD: superoxide dismutase
SPT: sucrose preference test
TST: tail suspension test
3 ′ UTR: 3 ′ untranslated region.
